This article has been retracted.

# Clinical Observation of MRI Image in Floating Needle Therapy for Cervical Spondylosis of Cervical Type

**DOI:** 10.1155/2022/1340192

**Published:** 2022-05-24

**Authors:** Xianqiang Liu, Zhenyi Tang, Botao Wang, Yongshuai Chen

**Affiliations:** ^1^Gradute School, Tianjin University of Traditional Chinese Medicine, Tianjin 301617, China; ^2^Department of Orthopedics, Tianjin Beichen Traditional Chinese Medicine Hospital, Tianjin 300400, China

## Abstract

In order to solve the problem of cervical spondylosis in the early stage of various cervical spondylosis, effective treatment can prevent the deterioration of the disease. This paper presents the results of a clinical trial examining magnetic resonance imaging in the treatment of cervical spondylosis with flotation therapy and selected 68 patients with cervical spondylosis. According to research commodity, using a rigorous randomized controlled trial, 34 cases were divided into a control group (acupuncture group). The needles were kept for 30 minutes once a day. The treatment group (acupuncture combined with floating acupuncture group) was treated with acupuncture on the 1st, 3rd, and 5th days and floating acupuncture on the 2nd, 4th, and 6th days, respectively. Both groups were treated for 6 consecutive days and rested for 1 day. After 2 weeks of treatment, the simplified McGill Pain Scale (MPQ), visual analogue scale (VAS), and neck pain scale (NPQ) were observed and recorded to compare the curative effects. Finally, Excel software is used to manage the data, and SPSS21.0 is used for statistical analysis. Measurements of gender, age, disease, VAS, simple MPQ, and NPQ of the two groups were compared in the two groups, *P* > 0.05, which was not significant and comparable. After treatment, VAS, simple MPQ, and NPQ of the two groups were compared in and between groups, the total *P* < 0.05, with the mean data. *Topics*. Acupuncture combined with float needle and acupuncture therapy can improve the pain and breathing of cervical spondylosis and improve the quality of life of patients, but acupuncture combined with needle float is more pronounced than acupuncture groups.

## 1. Introduction

Cervical spondylosis, tseem hu ua ligament joint capsule type cervical spondylosis, refers to a series of clinical syndromes caused by wind cold invading the local area; improper sleeping position or fatigue on the basis of acute and chronic injury of cervical muscles, joint capsule, and ligaments; dislocation of small joints; degeneration of intervertebral disc; and instability of vertebral body, resulting in excessive flexion or extension of cervical spine and compression or tension of some muscles, ligaments, or nerves in the neck. Most of the clinical manifestations are neck pain and limited activity. There are no obvious degenerative changes such as intervertebral space on X-ray films, but they can be accompanied by changes in cervical physiological curvature, vertebral instability, and mild hyperosteogeny. Most of them occur in the morning, the cold, or continuous fatigue, which is easy to ease naturally and occur repeatedly, and long-term repeated attacks will affect daily activities and quality of life. This type is very common in clinic and is the earliest stage of cervical spondylosis. In recent years, with the change of lifestyle, the number of long-term desk workers has increased, plus the incorrect posture of using the neck, resulting in the rising prevalence of cervical spondylosis, which has attracted more and more attention. The age of onset is also becoming younger. According to the survey, the incidence rate of cervical spondylosis among young and middle-aged is 19.22, while 29.1% of primary school students have abnormal cervical vertebra. This kind of patients' condition is light and heavy and easy to repeat, and many patients have insomnia, anxiety, and other symptoms. Some scholars believe that people with cervical spondylosis are prone to a lack of security and anxiety, which affects their physical and mental health. At the beginning of the disease, the symptoms are mild and transient, mainly local symptoms, and occasionally transient, which can be alleviated and easy to be ignored, which may develop into other types of cervical thrust disease. Cervical spondylosis is the first stage of various cervical spondylosis, and it is also the best time to treat and prevent other types of cervical spondylosis. Therefore, the treatment of cervical spondylosis is very important for the prevention and treatment of cervical spondylosis at all stages. At present, acupuncture has been widely used in the treatment of clinical NTCS. This treatment can effectively correct the block of Qi and blood along the meridians, so as to improve people's essence, Qi, and spirit, so as to achieve the purpose of treatment. In the treatment of clinical NTCS, acupuncture has significant advantages, not only because of its significant analgesic effect and less adverse reactions but also because it is a green therapy without any pollution. However, in the process of treatment, there are sometimes body position restrictions and more acupoints, which leads to some patients' resistance during treatment, which is easy to cause the end of treatment and reduce the therapeutic effect to a great extent. Therefore, it is necessary to evaluate treatment in combination with actual treatment effects to overcome the above limitations and make it easier for patients to improve health benefits. In recent years, a number of studies have confirmed that the occurrence and progression of NTCS are related to the muscles around the cervix, and the state of the muscles around the cervical spine plays an important role in the diagnosis of cervical spondylosis. As a new acupuncture physical therapy, floating acupuncture has the following advantages: There is obvious analgesic effect. The affected muscle can be transformed into normal muscle. There are less acupoints and convenient operation. The curative effect can be evaluated after each treatment. There are no restrictions on body position. And its indications are mainly the pain caused by muscle and soft tissue injury. The introduction of floating needle therapy into the treatment of NTCS can reperfuse the damaged muscles around the neck, so as to change muscle damage and spasticity, so as to improve the symptoms and signs of neck pain, neck stiffness, and limited activity, as shown in Figure 1.

## 2. Literature Review

Sheng-Lian and others said that cervical spondylosis (CS) refers to the syndrome with corresponding symptoms caused by the degeneration and proliferation of cervical intervertebral disc and various neck injuries or the prolapse of cervical intervertebral disc and the thickening of ligaments, which are squeezed into the adjacent spinal cord, cervical nerve, and cervical blood vessels [1]. Zheng and others think that according to the anatomical position of compression, it can be roughly divided into five types: nerve root type, vertebral artery type, spinal cord type, sympathetic nerve type, and neck type [2]. In recent years, Xu and others said that due to the rapid development of social economy, most people have changed in life, work, and learning methods, resulting in the incidence rate of spinal-related diseases being increased [3]. Xiao and others believe that this is due to the fact that the spine continues to maintain a fixed posture due to long-time sitting at the desk, resulting in the continuous fatigue of the whole spine, resulting in the occurrence of cervical spondylosis [4]. The incidence rate of incidence of cervical spondylosis is 3.8% and 17.6% and is related to occupation and age, with the incidence rate of 12%. Neck type cervical spondylosis (NTCS) belongs to the type with the lightest symptoms among all clinical types of cervical spondylosis. Its main clinical features are neck pain, neck stiffness, or limited activity. Me-Wu-Jia et al. said that the incidence rate of NTCS in the initial stage accounted for 40% to 60% of the total incidence rate of cervical spondylosis. If treatment is delayed or with improper treatment, it could develop into other types of cervical spondylosis. And studies showed that 80% to 90% of NTCS patients could be relieved of symptoms or even cured [5] by standard and systematic conservative treatment. Early prevention and treatment of NTCS are urgent. Ye and others said that cervical spondylosis belongs to the category of “arthralgia,” “neck and shoulder pain,” and “Xiang Qiang” in traditional Chinese medicine. There are various clinical treatment methods. Traditional Chinese medicine treatment includes oral administration, external application of traditional Chinese medicine, acupuncture, and massage, but most of them are comprehensive therapy [6]. Song and others think that acupuncture and moxibustion, as a green therapy, is widely accepted in clinic with better curative effect and less adverse reactions [7]. Xue and others said that in the process of clinical acupuncture treatment, doctors take more points and spend a long time on treatment, which not only increases patients' fear of acupuncture but also makes patients suffer a certain amount of pain in treatment [8]. The main methods of Western medicine treatment are symptomatic use of anti-inflammatory and analgesic drugs, physical therapy, and traction treatment. Its advantage is that it can alleviate symptoms relatively quickly, but with the recurrence of the disease, long-term use of analgesic and anti-inflammatory drugs will cause damage to liver and kidney function. Li and others said that in addition, incorrect operation of physiotherapy instruments or improper traction techniques may add additional pain to patients [9]. Yun and others feel that it is of great significance to explore a treatment scheme with convenient operation, rapid effect, and less pain [10]. Through the study of the experience of using a floating needle to treat various pain syndromes in clinic, it is observed that the floating needle has definite curative effect on the treatment of cervical spondylosis, especially in the change of pain degree after the first treatment, which greatly increases the patient's trust in doctors, and the number of times required for floating needle treatment is less than that of ordinary acupuncture, which greatly reduces the patient's pain. Therefore, based on the tutor's experience in the clinical treatment of cervical spondylosis with floating needle therapy, this time designs clinical trials, research methods, efficacy evaluation, and data management, so as to provide clinicians and patients with cervical spondylosis with a more effective, safe, and acceptable treatment scheme.

## 3. Method

Refer to the guidelines for diagnosis, treatment, and rehabilitation of cervical spondylosis (2010 edition) to determine the diagnostic criteria of cervical spondylosis: clinical symptoms: stiff neck and pain, which can stretch the whole shoulder and back in severe cases. In case of acute attack, you cannot do activities such as nodding, turning your head, and raising your head. When turning your head, you need to rotate together with your trunk, and your neck is in an oblique position. Clinical examination: nodding and head raising activities are not allowed in the acute stage, the activity of the cervical spine is absolutely limited, the range of activity of the cervical spine in all directions is close to zero, and there is multiple tenderness in the cervical muscle group. Common tenderness points are mostly located in T1~T7 paravertebral muscle, trapezius muscle, supraspinatus muscle, infraspinatus muscle, sternocleidomastoid muscle, etc. If there is secondary spasm of anterior scalene muscle, it can be on the inner side of sternocleidomastoid muscle, which is equivalent to the level of transverse process of neck 3-neck 6. Buckle it to the spasmodic muscle and press it with a little force, then there will be radiation pain in shoulder, arm, and hand. Imaging findings: the physiological curvature of cervical spine is slightly changed or normal, slight stenosis can be seen in intervertebral space, and hyperosteogeny can occur in some patients [11]. Clinical trials of traditional Chinese medicine refer to the clinical trials of cervical spondylosis in the Guidelines for Clinical Trials of New Chinese Medicines, some of which are included in the classification of cervical spondylosis. Syndrome of cold obstruction and collaterals: cold in the neck, stiff neck, dysfunction, fear of wind, cold and pain in the neck and shoulders, warm and appropriate [12], light red tongue, thin and white moss, and tight pulse string. Qi stagnation and blood addiction syndrome: it occurs due to neck trauma or injury, with strong pain in the neck, such as acupuncture, refusal to press the pain, fixed pain points, dark tongue, and astringent pulse strings. Liver and kidney deficiency syndrome: sore neck, increased fatigue, dizziness, shortness of breath, weak waist and knee, pale tongue, white fur, and heavy and weak pulse. The exclusion criteria were only abnormal imaging findings without clinical symptoms of cervical spondylosis, cervical spondylosis which is mainly of other types, no other serious systemic diseases, those who have obvious fear of acupuncture and refuse to cooperate with treatment, pregnant and lactating women who are allergic to acupuncture and have damaged skin, and observer who has received other analgesic treatment affecting the analgesic effect index of this trial [13]. The technology roadmap is shown in Figure 2.

Compressed sensing (CS) is a sampling method that can compress data proposed by Donoho. Traditional sampling generally uses the Nyquist sampling theorem, that is, Shannon theory, to discretize the signal. This theorem stipulates that the maximum frequency of a signal is Jmax, and when the minimum sampling frequency is greater than or equal to 2Jmax, the original signal can be restored without distortion through the sampling signal. However, with the rapid development of science and technology, the signal bandwidth is increasing day by day, and people's requirements for information processing speed are increasing day by day. The traditional sampling methods encounter great resistance in processing problems. The proposal of compressed sensing theory can well meet the existing sampling requirements, greatly reduce the operation cost, and improve the information processing speed, which provides a new sampling idea for signal processing [8, 14]. Finally, it is pointed out that the sparse signal can be reconstructed into a low-dimensional signal by using the theory of compressibility. From this assumption, it can be seen that signal density does not necessarily depend on bandwidth, which affects signal variability and inconsistency. Compressed sensing uses sampled and compressed signal features. The operation of compressed sensing is shown in Figure 3.

In Figure 3, the compressed sensing processing process mainly has three steps. In the first step, assuming that the input original signals *X*, *X* ∈ *R*^*n*∗1^ has sparsity on orthogonal bases *ψ* = [*ψ*_1_, *ψ*_2_, ⋯, *ψ*_*n*_] and *ψ*_*i*_ ∈ *R*^*n*∗1^, the compressed signal is shown in

(1) $$\begin{array}{c} S=\psi^{T}X. \end{array}$$

The second step is to select a matrix *Φ*, *Φ* ∈ *R*^*m*∗*n*^(*m*<<*n*) independent of the orthogonal basis and measure *s* linearly. The processing process is shown in

(2) $$\begin{array}{c} Y=\Phi S=\Phi \psi^{T}X=\Theta X, \end{array}$$

where Θ = *Φ*Ψ^*T*^,Θ ∈ *R*^*m*∗*n*^,*Y* ∈ *R*^*m*∗*n*^, we call Θ the sensing matrix. The original signal *s* is observed through the observation matrix *Φ* to obtain *m* observation values. Since *m* ≪ *n*, it is equivalent to transforming the high-dimensional signal into the low-dimensional signal. The third step is to solve the following objective function to obtain the reconstructed signal, as shown in

(3) $$\begin{array}{c} \arg\min\left\|\Psi^{T}X\right\|\\ \text{s}.\text{t}.\Theta X=\Phi S=Y. \end{array}$$

A sparse representation of a signal is the basis for compressed sensing applications. Only when the signal is small can it be guaranteed not to lose too much data after compression [15, 16]. The difference in the signal is easy to understand because there are few nonzeros in the signal, but the signal contained in the context is not complete, but approximately sparse in one exchange. In order to obtain different signal levels, it is important to find different representations. For any input signal *Y*, it can be expressed linearly as shown in

(4) $$\begin{array}{c} Y=\overset{n}{\underset{i=1}{\sum }}\varphi_{i}\sigma_{i}, \end{array}$$

where *φ*_*i*_ is a set of sparse basis vectors and *σ*_*i*_ is the transformation vector of *Y* in the phosphorus domain. If the sparse representation of signal *Y* requires at most *k* basis vectors and *K* ≪ *n*, the signal is said to be *k*-sparse. If most element values of vector *σ*_*i*_ are very small, the signal is said to be compressible. The traditional sparse representation of signals is mostly based on nonredundant orthogonal bases, such as wavelet transform, Fourier transform, and discrete cosine change. However, because the orthogonal bases required by different signals are different and different orthogonal bases have different characteristics, the use of a single orthogonal basis will have some limitations. For example, although wavelet transform can effectively represent point singular signals, it cannot well represent the high-dimensional function of line surface singularity, and Fourier transform cannot represent the characteristics of signals in time and frequency. In order to solve this problem, some researchers have proposed a signal sparse representation method based on combined orthogonal basis. In recent years, representations based on redundant dictionaries have also become a research hotspot. Redundancy dictionary refers to the complete redundant function, which is used to replace the basic function. This method can select the identity of the orthogonal basis according to the characteristics of the signal. At present, the sparse representation based on redundant dictionary is mostly studied from two aspects: the construction of redundant dictionary and the design of sparse decomposition algorithm. At present, there are two common sparse decomposition algorithms: matching pursuit and base pursuit. Matching pursuit (MP) is a sparse decomposition algorithm proposed by Mallat and others. It uses greedy algorithm to iteratively select the atoms that best approximate the signal structure from the Atomic Dictionary, but it is difficult to expand the signal after determining the selected atoms, because the atoms selected by the algorithm are not orthogonal to each other [17]. In order to solve this problem, Patl and others proposed orthogonal matching pursuit (OMP), which mainly realizes the signal expansion by orthogonalizing the selected atoms. The basis pursuit (BP) algorithm is proposed by Chen and others. It transforms the l0 norm minimization problem into the *H* norm minimization optimization problem, which can simplify the signal sparse decomposition process [18]. The selection of observation matrix *Φ* is very important for the realization of compressed sensing. Its quality directly affects whether the signal can be reconstructed correctly and whether the signal can be compressed to a great extent. This is because the main role of the observation matrix is to convert a high-dimensional signal to a low-dimensional signal without losing data, so that the signal velocity and the algorithmically constructed signal are based on the projection data, the first signal and observation matrices in low-dimensional space. A good observation matrix needs to meet the restricted isometric property rip condition, which stipulates that for any matrix *Φ*, if it satisfies the following formula, it is shown in

(5) $$\begin{array}{c} \left(1-\partial_{k}\right){\left\|X\right\|}_{2}^{2}\leq {\left\|\Phi X\right\|}_{2}^{2}\leq \left(1+\partial_{k}\right){\left\|X\right\|}_{2}^{2}. \end{array}$$

The matrix is said to meet the equidistant constraint, where *x* is the *k*-order sparse signal, *∂*_*k*_ is a constant, and the value range is (0, 1). Although the rip condition is of great significance, it is a necessary and insufficient condition, and it is impossible to directly verify whether the matrix meets this condition in practice. Based on this, Donoho and others proposed a more operable condition criterion, which stipulates that the observation matrix needs to meet the following conditions: the vector line of the observation matrix should be free and random; the vector line of the probe matrix must have some degrees of freedom, and the minimum value of the matrix containing it must be greater than the minimum value of the special matrix; the measured sparsity is in the *h*-norm minimal vector. The matrix meeting the above conditions can basically meet the rip condition; that is, it can be used as the observation matrix in compressed sensing. Common observation matrix construction methods include the following, based on orthogonal transformation, random sequence, binary matrix, specific signal, and polynomial. The specific introduction of each method is as follows. Based on the method of orthogonal transformation, this method mainly generates the observation matrix through the transformation of the orthogonal matrix. The specific steps are as follows: form an *N* × *N*-dimensional orthogonal matrix, then take *M* rows from the matrix to obtain an *M* × *N*-dimensional matrix, and finally, normalize the column direction of the matrix to obtain the observation matrix [19, 20]. At present, the observation matrix obtained by this method is mainly composed of the partial Fourier observation matrix and partial Hadamard observation matrix. This method is relatively simple and has certain stability, but there are still some disadvantages; that is, the partial Fourier observation matrix cannot reflect the characteristics in the time domain, there are certain limitations, and some Hadamard observation matrices have certain requirements for the length of signal and the number of observations. Signal reconstruction is simply to reconstruct the original signal 2 by using the observation sample *y* and the observation matrix *Φ*, that is, to solve the equation *y* = *Φx*. Since the number of observation samples is lower than the dimension of the original signal, there are countless solutions to the equation. However, because the compressed sensing theory requires that the original signal must be sparse, the above equation can be transformed into sparse solution by using this characteristic. The solution formula is shown in

(6) $$\begin{array}{c} \arg\min{\left\|x\right\|}_{0}\\ \text{s}.\text{t}.y=\Phi x. \end{array}$$

In formula (6), ‖*x*‖_0_ refers to the number of nonzero elements in the original signal. The model uses minimization. In theory, this method is feasible, but Donoho's research results show that to solve the above model, it is necessary to enumerate the arrangement of *C*_*N*_^*K*^ nonzero elements, which is a NP hard problem, so this method is not practical. After that, some researchers found that when the observation matrix is not related to the orthogonal basis, it can be solved by minimizing *l*_1_ norm instead of the above model. The formula is shown in

(7) $$\begin{array}{c} \arg\min{\left\|x\right\|}_{1}\\ \text{s}.\text{t}.y=\Phi x. \end{array}$$

In this way, an NP problem can become a problem solving problem, and further simplification can become a linear programming problem. As research progresses, scientists demand more signal recovery algorithms. Several decorations are shown below. Greedy algorithms are prepared by reducing technical knowledge. Because the latter belongs to the NP complex problem, the direct solution will waste a lot of time, so some scientists solve the problem in the past. The greedy algorithm uses only the signal coefficients and support settings to iteratively compute the best solution. The algorithm allows some errors in reconstruction. The advantage of the greedy algorithm is that it is fast and can be done in real time in practice, but the accuracy of the algorithm is low and requires high observations. In view of the shortcomings of this algorithm, many improved algorithms have been proposed, such as the orthogonal matching pursuit algorithm, compressed sampling matching pursuit CoSaMP, and stage wise orthogonal matching pursuit algorithm. A convex optimization algorithm solves the minimum *l*_1_ norm to reconstruct the original signal. This algorithm is also proposed to solve the problem of minimizing *l*_0_ norm. It is found that when the observation matrix is not related to the orthogonal basis, the problem of minimizing *l*_0_ norm can be transformed into the problem of minimizing *l*_1_ norm; that is, it becomes a convex optimization problem. Finally, the original signal can be reconstructed by linear programming. The algorithm has the advantages of high precision and less observations, but it is not suitable for processing large-scale signals, and the running time of the algorithm is long. In addition, its search direction is easily affected by the observation matrix, so it is necessary to reasonably select the observation matrix for the algorithm. At present, common convex optimization algorithms include base tracking algorithm, gradient projection for sparse reconstruction (GPSR), and iterative hard threshold algorithm (IHT) [21]. The statistical optimization algorithm first generates a training set with the help of typical signals, then finds the optimal linear projection set through a certain learning algorithm, and finally uses the set to reconstruct the signal. Although the algorithm requires more observations than the convex optimization algorithm, it takes less time to run, which can achieve a good balance between the two. At the same time, the accuracy of the algorithm is high [22]. At present, the common statistical optimization algorithms are the algorithm based on Bayesian statistics and the statistical optimization algorithm based on training set learning. The combination algorithm mainly uses highly structured and group testing to obtain the support set of the signal. Compared with the convex optimization algorithm, it runs faster and requires less observations. However, the combination algorithm does not specifically limit the observation matrix, which makes it difficult to propose a new observation matrix. In addition, the accuracy of the algorithm cannot be fully guaranteed [23, 24]. At present, the more popular combination algorithms include chain pursuit (CP), Fourier sampling, and HHSP (heavy hitters on steroids pursuit). Signal reconstruction is very important in the process of compressed sensing. The error of the original signal reconstructed determines the performance of compressed sensing. At present, a large number of signal reconstruction algorithms have been proposed, but these algorithms still have some limitations. Therefore, how to obtain reconstruction algorithms with low time complexity and high precision is still a difficult and hot spot for researchers to solve. A compressed tracking algorithm is a robust tracking algorithm based on compressed sensing theory. It is simple and efficient and has been used in many fields. Compressed sensing theory points out that a random matrix satisfying the condition of compressed isometry property rip is used to randomly sample the sparse vector, and the sampled low-dimensional vector retains almost all the information of the original vector. CT algorithm samples and compresses high-dimensional features according to this theory, and its tracking process is shown in Figure 4.

Haar-like feature is used here. Haar-like feature is a common feature description operator in the field of computer vision. It uses a random matrix *E* with dimension *M* × *N* satisfying rip conditions to convert the high-dimensional feature vector *X* (*n*-dimensional) to the low-dimensional feature vector *V* (*m*-dimensional), where *m* is much less than *n*. The formula is shown in

(8) $$\begin{array}{c} V=EX. \end{array}$$

The random matrix *e* is a very sparse matrix, and the values of the elements in row *Z* and column *J* are shown in

(9) $$\begin{array}{c} e_{i,j}=\sqrt{s}*\left\{\begin{array}{cc} 1, & \text{the probability is }{\left(2s\right)}^{-1},\\ 0, & \text{the probability is }1‐s^{-1},\\ -1, & \text{the probability is }{\left(2s\right)}^{-1}. \end{array}\right. \end{array}$$

When *s* = *O* (*n*), matrix *E* satisfies the rip condition, and at most four nonzero elements in each row need to be calculated, which can effectively improve the running speed of the algorithm. The CT algorithm uses the naive Bayesian classifier for classification and uses formula (8) to obtain the low-dimensional feature vector *V* = (*v*_1_, ⋯,*v*_*m*_)^*T*^ of the sample image. Assuming that the components in the feature vector are independent of each other and the probability that each sample is a target or background is the same, the model of naive Bayesian classifier is shown in

(10) $$\begin{array}{c} H\left(v\right)=\overset{m}{\underset{i=1}{\sum }}\log\left(\frac{p\left(v_{i}\right.\left|y=1\right.}{p\left(v_{i}\right.\left|y=0\right.}\right). \end{array}$$

When evaluating treatment outcomes, carefully consider any adverse or unexpected events (including the patient's symptoms and signs) and cause, make similar decisions, and write them down. In serious cases, the exam will be cancelled. For adverse events in the experiment, symptoms, signs, degree of occurrence, time of occurrence, timing, treatment, etc., shall be recorded on the case report form to evaluate their correlation with the test methods and acupoint selection, which shall be recorded in detail by the researcher, who shall sign and indicate the date of the event [25]. The possible adverse events in this test mainly include needle fainting, hematoma, and infection caused by the retention of floating needle hose. Judge the relevant conditions of adverse events in detail, such as occurrence time, main symptoms, duration, severity, treatment measures taken, and disappearance time. After evaluating the adverse reactions, judge whether to terminate the test according to the severity of the situation. According to the adverse reactions of different cases in this study, determine the safety classification and then count the number of cases in each safety classification of different treatment schemes. After statistical analysis, the safety of different treatment schemes can be evaluated [26]. The safety evaluation is graded as follows: Level 1: safe without any adverse reactions. Level 2: relatively safe, with adverse reactions, but to a lesser extent, and the treatment can be continued without any treatment. Level 3: safety concerns and adverse reactions. Degrees are average. Treatment can be continued after symptoms are treated. Grade 4: the study was postponed due to adverse reactions.

## 4. Experiment and Analysis

A total of 70 eligible studies were included in this study, including 35 cases in the experimental group and 35 cases in the control group. Among them, 3 cases were lost to follow-up due to personal reasons, and no circumstances were excluded. The final treatment included 34 cases in the experimental group and 32 cases in the control group, a total of 66 cases. See Table 1 for the completion status.

In the process of this study, there were 4 cases of abscission, and no cases were excluded, accounting for 4.41 of the total design samples. Among them, 1 case fell off in the floating needle group and 3 cases fell off in the conventional acupuncture group. The difference between the groups was not statistically significant by the *χ*^2^ test, *P* > 0.05. Case rejection/shedding is shown in Table 2.

Three cases did not complete the treatment plan, including 2 cases of noncompliance with the treatment due to occupation (4 cases in the treatment group and 7 cases in the control group) and 1 case of noncompliance, seeing a doctor due to inconvenience of transportation. The other cases were successfully treated according to the trial design steps, and the completion rate was 95.59%. The gender comparison between the two groups is shown in Table 3.

According to the statistical analysis of the gender distribution of the subjects in the test group and the control group, the *χ*^2^ test shows that *χ*^2^ = 0.365, *P* = 0.524 > 0.05, so the gender distribution difference between the two groups is not statistically significant and comparable. The age comparison between the two groups is shown in Table 4.

The oldest in the medical group was 52 years old, and the youngest was 21 years old. On the board of directors, the oldest is 51 years old and the youngest is 25 years old. The age comparison of the two groups and the face test showed that *t* = −0.123, *P* = 0.903 > 0.05; the difference was not significant and significant. The comparison of the two groups of diseases is shown in Table 5.

The data did not follow a normal distribution after natural measures analysis compared to the disease categories of the two groups, so two independent examples without the use of a test (Mann-Whitney *U* test) were used. The test results showed that *Z* = −0.539, *P* = 0.590 > 0.05, the difference was not significant, and the two groups were compared. The comparison of symptoms between the two groups is shown in Table 6.

There was no significant difference in the distribution of TCM syndromes between the two groups (*P* > 0.05). After the first course of treatment and one course of treatment, the VAS scores of both groups were lower than those before treatment. Two discordant samples (Wilcoxon sign test scale) differed significantly (*P* < 0.05): test VAS scores after the first treatment compared with both groups. From the two noninvasive tests (Mann-Whitney *U* test), the difference was significant; after one course of treatment, the VAS scores of the two tests were not inconsistent (Mann-Whitney *U* test); the difference was not significant (*P* > 0.05), as shown in Figure 5.

Cervical spondylosis is the highest incidence rate in all types of cervical spondylosis, accounting for 4086. In recent years, with the incidence rate of cervical spondylosis increasing, the age of onset of cervical spondylosis is gradually younger. Therefore [27], many doctors are trying to explore in clinic to find a way to relieve pain and be convenient, simple, safe, nontoxic, and effective. Acupuncture and moxibustion therapy are the most widely used intervention for cervical spondylosis of cervical type. The accuracy and safety of its efficacy have been confirmed by a large number of clinical applications and studies. Therefore, this study takes the conventional acupuncture group as the control group to explore the clinical application advantages of floating acupuncture therapy. Floating needle therapy is a new acupuncture technology invented by Professor Fu Zhonghua based on Ashi point theory and wrist manic needle theory. Because of its significant analgesic effect and convenience of operation, it is widely used by clinical doctors to treat various bone injuries, pain diseases, and medical miscellaneous diseases, especially for pain caused by muscle and soft tissue injury. The analgesic effect is immediate. Therefore, by comparing the overall efficacy, immediate analgesic effect, and impact on emotional life of acupuncture and floating needle therapy in the intervention of cervical spondylosis, this paper comprehensively analyzes the advantages of floating needle therapy, so as to provide guidance and basis for its further wide application in clinic.

## 5. Conclusion

In overall evaluation, acupuncture is based on the theory of Yu acupoints in the meridians, “the meridians pass through and the main treatment reaches,” which plays a role in harmonizing Yin and Yang and dredging the meridians, so as to treat NTCS. Acupuncture plays an irreplaceable role in the treatment of NTCS and is widely used in clinic. In the treatment of NTCS, a floating needle mainly selects the affected muscle, which makes the target more accurate and avoids the disadvantage of blind selection. Moreover, the selection of points by floating needle is less than that by conventional acupuncture, which reduces the physical and mental pressure of patients to a certain extent. The floating needle has the advantages of quick effect and nontoxic side effects. In general, floating needle therapy has comprehensive advantages in the treatment of NTCS. Therefore, this study chose the complementary way of floating needle therapy and acupuncture therapy to improve the overall curative effect. This study combines the pathogenesis characteristics of NTCS and follows the principle of tendon disease following meridians, so as to achieve the purpose of treating NTCS. Both floating acupuncture and conventional acupuncture can effectively improve the pain symptoms of cervical spondylosis, and the curative effects of both are equivalent. After the first treatment, floating acupuncture was significantly better than conventional acupuncture in improving the degree of pain, indicating that floating acupuncture has better immediate analgesic effect. Under the condition of considerable clinical efficacy, safety, and compliance, the number of treatment times required by floating needle is less than that of conventional acupuncture, which is conducive to reducing the pain of patients, saving the time cost of doctors and patients, and improving clinical efficiency.

## Figures and Tables

**Figure 1:** Clinical observation of image in floating needle therapy in the treatment of cervical spondylosis of cervical type.

**Figure 2:** Technical circuit diagram.

**Figure 3:** Compressed sensing processing flow.

**Figure 4:** Basic flow of compression tracking.

**Figure 5:** VAS score comparison.

**Table 1:** Completion of two groups of cases.

Group	Number of cases	Removal/shedding	Complete
Treatment group	35	1	34
Control group	35	3	32
Total	70	4	66

**Table 2:** Summary of case rejection/shedding.

Group	Number	Removal/shedding	Reason	Time
Treatment group	12	1	Work	4th time
Control group	3/25	2	Inconvenient transportation	7th time

**Table 3:** Comparison of gender composition between the two groups.

Group	Number of cases	Male (%)	Female (%)
Treatment group	33	16 (48.5%)	17 (51.5%)
Control group	32	17 (53.1%)	15 (46.9%)

**Table 4:** Age comparison between the two groups.

Group	Number of cases	Average age (years)	*t*	*P*
Treatment group	33	33.39 ± 8.5	-0.123	0.903
Control group	32	33.63 ± 6.4		

**Table 5:** Comparison of course of disease between the two groups (*x* ± *s*, month).

Group	Number of cases	Average course of disease (months)	*Z*	*P*
Treatment group	33	3.70 ± 1.45	-0.53	0.59
Control group	32	3.88 ± 1.29		

**Table 6:** Comparison of syndrome types between the two groups.

Group	Number of cases	Wind cold blocking collaterals	Qi stagnation and blood stasis	Deficiency of liver and kidney
Treatment group	33	10	17	6
Control group	32	9	16	7

## Data Availability

The data used to support the findings of this study are available from the corresponding author upon request.
